This article has been retracted.

# Gypenosides regulate autophagy through Sirt1 pathway and the anti-inflammatory mechanism of mitochondrial autophagy in systemic lupus erythematosus

**DOI:** 10.1080/21655979.2022.2066749

**Published:** 2022-06-05

**Authors:** Jin-Yong Ke, Zhi-Yong Liu, Yun-Han Wang, Shi-Ming Chen, Jing Lin, Fang Hu, Yu-Fang Wang

**Affiliations:** a Department of Hematology, Huangshi Central Hospital, Edong Healthcare Group (Affiliated Hospital of Hubei Polytechnic University), Huangshi, Hubei, China; b Department of Rheumatology, Huangshi Central Hospital, Edong Healthcare Group (Affiliated Hospital of Hubei Polytechnic University), Huangshi, Hubei, China; c Department of Rheumatism Immunity, Renmin Hospital of Wuhan University, Wuhan, Hubei, China; d Guangzhou University of Chinese Medicine, Guangzhou, Guangdong, China; e Department of Clinical Laboratory, Huangshi Central Hospital, Edong Healthcare Group (Affiliated Hospital of Hubei Polytechnic University), Huangshi, Hubei, China

**Keywords:** Gynostemma pentaphyllum saponins, systemic lupus erythematosus, Sirt1 pathways, mitochondrial autophagy

## Abstract

To study the mechanism of *gynostemma pentaphyllum* saponins (GpS) regulating mitochondrial autophagy and anti-inflammatory through Sirtuin 1 (Sirt1) pathway in systemic lupus erythematosus (SLE). JURKAT cells were cultured in vitro, RT-PCR and western blotting (WB) were utilized to identify the expression of related-proteins in Sirt1 pathway and global autophagy and mitochondrial autophagy markers in JURKAT before and after GpS treatment induced by ultraviolet B (UVB), and the related-mechanism of GpS regulation of autophagy was analyzed. The SLE model was established to analyze the alleviating effects of GpS on various symptoms of lupus mice. Sirt1/AMPK/mTOR pathway was activated in UVB induced JURKAT cells. After the addition of GpS, WB revealed that the phosphorylation of AMPK decreased, the phosphorylation of mTOR increased, the expression of Sirt1 protein decreased, and the activation of the pathway was inhibited. Moreover, autophagy of JURKAT cells wasinhibited. In order to further verify the role of Sirt1 pathway, we activated Sirt1 expression in cells by constructing lentiviral vectors, and the therapeutic effect of GpS was significantly reduced. These results indicate GpS can exert autophagy regulation by inhibiting the activity of Sirt1 pathway. To treat SLE. GpS can significantly reduce the level of autoantibodies, kidney inflammation, immune complex deposition and urinary protein excretion, improve kidney function in lupus-prone mice. GpS can regulate autophagy and mitochondrial autophagy through Sirt1 pathway, which may be a potential mechanism for GpS to reduce the level of autoantibodies, kidney inflammation, immune complex deposition and urinary protein excretion, improve kidney function in lupus-prone mice.

## Highlights

- GpS can regulate autophagy and mitochondrial autophagy through Sirt1 pathway;
- GpS to reduce the level of autoantibodies, reduce kidney inflammation and immune complex deposition;
- GpS to improve kidney function, and reduce urinary protein excretion in lupus-prone mice.

## Introduction

Systemic lupus erythematosus (SLE) is a representative systemic autoimmunity illness. Complicated interactions of damaged amphoteric body space, innate and adaptive immune system regulation, supplemental activation, immune complexes and tissue inflammation ultimately lead to self-sustaining autoimmune process [1,2]. There is a significant burden of disease among different races, races and age groups around the world [3].

Sirtuin 1 (Sirt1) is responsible for the encoding of one member of the sirtuin protein family, which is homologous to the yeast Sir2 protein. Such genetically encoded proteins belong to class I of the sirtuin family. Variable splicing leads to several transcriptional mutations [4]. The components of the sirtuin family are featured by the core domain of sirtuin and are divided into four categories. The functions of mankind sirtuins haven’t been identified yet. Nevertheless, sirtuin protein modulates epigenesis genetic silencing and inhibit recombinant rDNA [5]. Researches have shown that mankind sirtuins might act as endocellular modulatory protein with single ADP ribose transferase activity [6]. Sirt1 is turning into a pivotal target for novel treatments of a variety of illnesses, such as inflammatory diseases and autoimmunity diseases [7,8]. Hu et al. [9] discovered that Sirt1 over expression is related to the etiopathogenesis of SLE, and the down-regulation of Sirt1 alleviated the injury in SLE. Coniglio et al. discovered that Sirt1 can change the incidence of SLE in south Brazil [10]. It is noticeable that Sirt1 takes an important part in the regulation of many biological functions including cell autophagy. Sirt1 could promote autophagy and inhibits apoptosis to protect cardiomyocytes from hypoxic stress [11]. A body of studies has confirmed that resveratrol treatment protected osteoblasts in osteoporosis rats by enhancing mitophagy through mediating SIRT1 signaling pathway [12]. Nevertheless, its causal link of the onset and progression of SLE is still unclear.

Autophagy is a process in which cells wrap some of their own proteins or organelles in a specific membrane structure and transport them to lysosomes for degradation, producing energy and nutrients for repeated use by cells [13]. Autophagy not only provides energy for cells and maintains cell homeostasis, but is also closely related to the immune system. If the regulation of autophagy is abnormal, it will lead to the occurrence of autoimmune diseases, such as SLE. Studies have shown that the level of autophagy in SLE is increased, and Disease activity is related [14]. Autophagy can not only regulate cells, but also regulate signal pathways to activate or inhibit them [15]. In addition, mitochondrial autophagy is a special form of selective autophagy, which refers to the process in which excess or damaged mitochondria can be selectively eliminated by cells through the autophagy mechanism [16]. Although the understanding of the molecular mechanism of autophagy has been greatly expanded in recent years, a large amount of further evidence is still needed to establish a comprehensive clinical environment and target the autophagy pathway of SLE patients. The study of the role of autophagy in SLE pathology, especially in organ pathology, is still a largely under-researched area.

At present, patients with SLE are usually treated with immunosuppressants and glucocorticoids [17]. The development of SLE treatment is limited by clinical and biological heterogeneity, including the diversity of peripheral blood gene expression characteristics [18]. Recently, naturally formed products have received increasing attention due to their minor side effects. In view of their effective biological activity and good health benefits, they can be used to prevent and treat certain diseases. *Gynostemma pentaphyllum* saponins (GpS) are extracted from *Gynostemma*, and many pharmacological effects of *Gynostemma* have been reported in recent years, such as anti-cancer, anti-ulcer, treatment of hepatitis and hyperlipidemia [19]. Studies have also found that GpS has therapeutic potential in atherosclerosis by enhancing Sirt1-FOXO1-mediated autophagic flux recovery, inhibiting ox-LDL uptake and foam cell formation [20]. However, there is currently no research report on the treatment of GpS in SLE.

In view of the important role of Sirt1 in SLE, the aim of this study was to explore the effect of GpS on SLE and clarify the underlying molecular mechanisms. GpS might play treatment roles in SLE, and it acts on the Sirt1 pathway to regulate the overall autophagy level of SLE to exert immune regulation. effect. We will also study the effect of GpS on the level of mitochondrial autophagy in SLE to unravel the causal link of GpS in the SLE therapy.

## Materials and methods

### JURKAT cell cultivation

JURKAT cells (Stem Cell Bank of CAS) were added to the complete culture medium: RPMI1640 medium with 10% FBS and 1% penicillomycin antibiotics, and cultivated in an incubating device at 5% carbon dioxide under 37°C. Subculture or subsequent experiments were conducted when the cells reached 70–90% confluence (logarithmic growth phase).

### MTT method to detect cell viability

JURKAT cells (Stem Cell Bank of CAS) at logarithmic growth stage were selected, digested with 0.125% trypsin, and conventionally inoculated into 96-well plates. The cells (5 × 10^3^) were cultured at 37°C temperature with 5% CO_2_ for about 1–2 days. When the cell confluence observed under the microscope reached 70–90%, drugs with gradient concentration (0, 2, 5, 10, 20, 40, 80 μM) were added to make the final volume of each well 100 μL. About 10 μL MTT (5 mg/mL) was added to each well (Thermo Fisher Scientific, Shanghai, China), and placed in an incubator for continued operation for 4 h. The absorbance value at 570 nm was measured and the corresponding curve was drawn.

### Cell transfection

JURKAT cells at logarithmic growth stage were infected with lentivirus-packed plasmids encoding Sirt1 protein to establish JURKAT cell lines expressing Sirt1 stably.

### qRT-PCR assay

Overall RNA was extracted via TRIzol reagent (Sigma-Aldrich, America). Reverse transcript of RNA was performed using ReverTra Ace qPCR RT Tool (Toyobo Life Science, Japan). FastStart Universal SYBR Green Master (Roche Applied Science, Germany) was utilized for transcription, GAPDH was used as internal reference, and expression quantity was calculated using 2−∆∆Ct method. The primer sequence was as follows: AMPK forward: 5'- TCTGAGGGGCACCAAGAAAC-3', reverse: 5'-GTGGGTGTTGACGGAGAAGAG-3'; Sirt1 forward: 5'- TAGCCTTGTCAGATAAGGAAGGA-3', reverse: 5'- ACAGCTTCACAGTCAACTTTGT-3', mTOR forward: 5'- GCTAGGTGCATTGACATACAACA −3', reverse: 5'- AGTGCTAGTTCACAGATAATGGC-3'; ATG7 forward: 5'- ATGATCCCTGTAACTTAGCCCA-3', reverse: 5'- CACGGAAGCAAACAACTTCAAC-3'; Beclin-1 forward: 5'- GCCCAGACAGGACTCTCTTAG-3', reverse: 5'- TGAACACACTTGCCAGTCTTC-3'; LC3 II forward: 5'- CCCAAGCGTCAGACCCTTC-3', reverse: 5'- GGGGAACTTTGCCCGGATT-3'; TOMM20 forward: 5'- TGTATTTACCTCAACCGGAAGC-3', reverse: 5'- TCGCACACTAAAAGGGCATTG-3'; TIM23 forward: 5'- GAAGGTGGCGGAAGAAGTAGC-3', reverse: 5'- GGGGGTTCATACCAGTCAGC-3'; GAPDH forward: 5’-TGTGGGCATCAATGGATTTGG-3’, reverse 5'- ACACCATGTATTCCGGGTCAAT −3'; U6 forward: 5’- GATTATCGGGACCATTCCACTG-3’, reverse 5'-GATCTGGTTCCCAATGACTGTG-3'.

### Immunoblotting assay

The cells were subjected to homogenization in RIPA protein lysis buffering solution with protease suppressor for 30 min and then centrifuged at 12,000 g under 4°C for 20 min. The protein level was identified via the BCA protein analysis tool (Pierce, Rockford, IL, USA). Total protein was loaded onto 10% SDS-Page (Beyotime, Shanghai, China) and moved onto polyvinylidene fluoride (PVDF) film (Millipore, America). The membrane was blocked via 5% skin milk for 2 h and afterward incubated overnight at 4°C with corresponding the primary antibodies (Abcam, Cambridge, MA, USA). After that, the membrane was washed 3 times in PBST and incubated for 2 h with secondary antibodies (Abcam, Cambridge, MA, USA), cleaned 3 times in poly(butylene succinate- co-butylene terephthalate) (PBST), and then analyzed by electrochemiluminescence (ECL) and image analysis program (NIH, America). *β*-actin was utilized as control.

### UVB radiation

UVB irradiation method [21]: Irradiation time (s) = required irradiation measurement/emitter intensity. Irradiation distance 5 cm. The dose was 50MJ /cm^2^. UVB irradiation instrument (SS01B-2) was purchased from Shanghai Sigmar High Technology Co., LTD.

### JC-1 dyeing to identify variations in cell MMP (ΔΨm)

The cells digested by trypsin were inoculated at 2 × 10^5^ cells per well in a cell culture box with 5% CO_2_ at 37°C. When the cell density reached about 80%, 6 ml JC-1 staining solution was diluted in 6 ml fresh cell culture solution, and fully mixed, 2 ml was added to each well at 37°C. Incubated in 5% CO_2_ cell culture box for 20 min; after incubation, discard the supernatant and wash it with JC-1 staining buffer for 3 times. 2 ml cell culture medium was added to each well and observed under fluorescence microscope: When ΔΨm was high, JC-1 would form polymer in the mitochondria substrate and generated red fluorescent result. When ΔΨm is low, JC-1 is monomer and generates green fluorescent result.

### Experimental animals

Healthy female MRL/LPR lupus-prone mice, 6–8 weeks, 20–22 g, 7 mice per group, bought from Slyke Lab Animal Co., LTD. The experimental animals were fed and watered freely and kept at room temperature 18–23°C. The feed and pad materials were bought from the Experiment Animal Center of CMU. Through UVB induced disease progression, the present research was accepted by the Ethical Board of our hospital.

### Mouse urine collection

During the feeding process, metabolized urine of mice was collected in a mouse metabolic cage for 12 hours per week. After centrifugation, the urine was placed in a 1.5 mL EP tube and stored at −80°C. Urine protein content was determined by Bradford method [22].

### Mouse serum collection

After taking blood from eyeballs, the mice were sacrificed. First, mice were subjected to anesthetization via 10% chloral hydrate (0.08 mL/mouse). Next, the whiskers were clipped to prevent hemolysis, and one of the eyeballs was clipped with tweezers to allow the blood to flow into a 1.5 mL centrifuge tube. The specimens were placed under RT for about 60 min, subjected to centrifugation under 1500 RPM for 600 s at 4°C. The upper serum was extracted and stored at −80°C.

### Collection and retention of mouse kidney tissue samples

The animals were sacrificed by cervical dislocation. Skin tissue was slowly stripped, the whole thorax was exposed, blood vessels were separated, and kidneys were removed. It was completely immersed in 4% paraformaldehyde solution, fixed for 72 h, then dehydrated with alcohol gradient, embedded with paraffin embedding technology, used for renal tissue section. Renal tissue sections were used for H&E staining.

### Immunofluorescence staining

After paraffin sections of kidney tissue were baked, dewaxed and rehydrated, washed three times in cold PBS, blocked with 5% goat serum for 1 h. Next, sections were incubated with primary antibody overnight at 4°C. After night, under RT for 60 min, the PBS solution was cleaned three times, 10 min/time, and the PBS outside the specimen was wiped with filter paper. After that, the corresponding immunofluorescence secondary antibody 50 µl was dropped and stood for 2 h at room temperature, protected from light. After the second antibody was incubated for 2 h, the PBS solution was cleaned three times, 10 min at a time, and the excess PBS was erased with filter paper. The tablets were sealed with DAPI, and immediately observed under a fluorescence microscope and photographed at magnification ×200.

### Immunohistochemical method

The tissue was fixed in 4% paraformaldehyde fixative solution (4°C). After fixation, the tissue was washed with PBS for 3 times, and the tissue was placed in ethanol for gradient dehydration (4°C). After that, the tissue was placed in liquid paraffin. Poly-l-lysine was soaked in 3% hydrogen peroxide to inactivate endogenous enzymes. The slices were immersed in 0.01 M citrate buffer, heated to boiling, repeated twice after 5 minutes, and washed with PBS after cooling. Added 5%BSA block solution for 20 min at room temperature, added primary antibody at 37°C for 1 h, and washed with PBS. Added secondary antibody, incubating at 37°C for 20 min, and washed with PBS. DAB color kit was used for room temperature coloration, washed with distilled water, and finally mildly restained with hematoxylin, differentiated with alcohol hydrochloric acid, rinsed with distilled water, dehydrated and dried with gradient alcohol, transparent with xylene, sealed with neutral gum, and observed under a microscope.

### Autoantibody detection

Alpha Diagnostic International (ELISA) was employed to identify the expression levels of IFs, such as IL-1, IL-1β, IL-6, IL-10, TGF-β and IFN-γ, in renal tissues. For details, refer to the kit specification.

### Statistics

The entire statistic assay was completed via GraphPad Prism 6.01, and the outcomes were mean ± SD. The diversities between these groups were studied via a one-way ANOVA method, and the Tukey test was used to correct for multiple comparisons. The students’ test was employed to contrast the two groups. *P*< 0.05 has significance on statistics.

## Results

The current study is designed to determine the effect of GpS on SLE and clarify the underlying molecular mechanisms. GpS might play treatment roles in SLE, and it acts on the Sirt1 pathway to regulate the overall autophagy level of SLE to exert immune regulation. effect. We also investigate the effect of GpS on the level of mitochondrial autophagy in SLE to unravel the causal link of GpS in the SLE therapy.

### The concentration and time of GpS action on JURKAT cells were determined by MTT method

In order to determine the working concentration of GpS, JURKAT cells were exposed to diverse levels of GpS for 6 h, and the cellular activity was identified via MTT method, and the cell viability curve was drawn. The concentration of GpS was selected based on the maximum concentration of GpS without causing a decrease in cell viability. Therefore, the working concentration of GpS was selected as 40 μM. (Figure 1)

**Figure 1.** Cellular activity of JURKAT cells with diverse levels of GpS. *P< 0.05.

### GpS inhibited the activation of Sirt1 pathway in JURKAT cells

We treated JURKAT cells with UVB and UVB+GpS for 6 hours and then extracted proteins, and detected related pathway proteins by RT-PCR and western blotting. We found that under the induction of UVB, the Sirt1 pathway of JURKAT cells showed an activated state: the content of Sirt1 and p-AMPK increased, and the content of p-mTOR was reduced (P < 0.05). In the UVB+GpS group, in contrast to the UVB one, the levels of Sirt1 and p-AMPK decreased, and the level of p-mTOR was elevated (P < 0.05). The above results reflect that GpS plays a role by inhibiting the activity of Sirt1 pathway (Figure 2).

**Figure 2.** GpS inhibits activation of Sirt1 pathway in JURKAT cells. A: PCR detects the expression level of Sirt1 pathway genes in cells. B: Western blotting detects the expression level of Sirt1 pathway protein. *P< 0.05.

### GpS inhibited the autophagy related genes and proteins level of JURKAT cells

RT-PCR and western blotting analyses were employed to identify the expressing levels of autophagy related proteins and genes. As shown in Figure 3, after GpS was added, the contents of ATG7 mRNA, Beclin-1 mRNA, LC3 II mRNA, ATG7, Beclin-1 and LC3 II decreased. Autophagy activity was reduced (P < 0.05), indicating that GpS may play a important role in the overall autophagy level of cells.

**Figure 3.** GpS inhibits the overall autophagy level of JURKAT cells. A: PCR detects the expression level of autophagy genes. B: Western blotting detects the expression level of autophagy protein. *P< 0.05.

### GpS inhibited mitochondrial autophagy in JURKAT cells

In order to further explore the mechanism of GpS, we chose the entry point of mitochondrial autophagy and mitophagic activities for research. Mitochondrial content was measured by mitochondrial outer membrane protein TOMM20 and mitochondrial inner membrane protein TIM23. After PCR and Western blotting, we found that the levels of TOMM20, TIM23 and δ ψ M decreased after UVB irradiation, while the levels of these three indexes increased with the addition of GpS (P < 0.05).

To examine the changes in mitochondrial function more closely and determine whether UVB induces abnormal activation of mitochondrial autophagy, and whether GpS inhibits the occurrence of mitochondrial autophagy. Mitochondrial autophagy means that mitochondria are surrounded by a bilayer membrane formed by the fusion of autophagic lysosomes. UVB reduces the number of mitochondria and promotes the formation of autophagic vesicles containing mitochondria (intact or almost degraded). GpS alleviates the UVB-induced decrease in the number of mitochondria and inhibits the formation of autophagic vesicles surrounding mitochondria. We used PCR and western blotting to evaluate the changes in mitochondrial autophagy. Our results indicated that UVB irradiation increased the mRNA and protein levels of ATG7, Beclin-1 and LC3 II (Figure 4c, d). The above results showed that GpS inhibited mitochondrial autophagy in JURKAT cells (Figure 4).

**Figure 4.** GpS inhibits mitochondrial autophagy in JURKAT cells. A, B: Detection of mitochondrial content. C: PCR detects the expression level of autophagy genes. D: Western blotting detects the expression level of autophagy protein. E: Changes in mitochondrial membrane potential. *P< 0.05.

### Activation of Sirt1 pathway significantly inhibited the effect of GpS

We also found that GpS remarkably suppressed the expressing of Sirt1 in JURKAT cells, and the expression of AMPK was also decreased, while the expression of mTOR was increased. In order to verify the role of Sirt1/AMPK/mTOR signaling pathway, we overexpressed Sirt1 expression in JURKAT cells by constructing lentiviral vectors, at which AMPK expression was elevated and mTOR expression was inhibited (P < 0.05), and significantly inhibited the effect of GpS, and the levels of TOMM20, TIM23, and δ ψ M decreased (P < 0.05). These results suggest that GpS inhibits mitochondrial autophagy in JURKAT cells by inhibiting Sirt1/AMPK/mTOR signal path (Figure 5).

**Figure 5.** Activation of the Sirt1 pathway significantly inhibits the effect of GpS. A: The effect of GpS on the gene expressing of Sirt1/AMPK/mTOR signal path. B: The effect of GpS on the protein expressing of Sirt1/AMPK/mTOR signal path. C: Verification of the transfection effect of the lentiviral vector. D: Detection of mitochondrial content. E: Changes in mitochondrial membrane potential. *P< 0.05.

### GpS reduces kidney inflammation in lupus-prone mice

Renal histopathology confirmed that mice in the Model group showed severe renal injury characterized by extensive inflammation cell infiltration, partial glomerulosclerosis, visible crescent formation, enlarged mesangial stroma, and diffuse perivascular and interstitial inflammation cell infiltrating. In the treatment group, glomerular inflammatory cell infiltration, glomerulosclerosis, interstitial and perivascular lesions were significantly reduced (*P*< 0.05), HE staining results showed that compared with Model, glomerular and tubule scores were lower in GpS feeding group (*P*< 0.05) (Figure 6a), and with the treatment of GpS, the expression of Sirt1 in cells decreased significantly

**Figure 6.** GpS can reduce kidney inflammation in lupus-prone mice. A: HE staining score. B: Immunohistochemical results of Sirt1 in each group. C: ELISA to detect the level of inflammatory factors. *P< 0.05.

(Figure 6b). ELISA results also showed that GpS significantly inhibited renal tissue inflammation in mice (*P*< 0.05) (Figure 6c).

### GpS reduced serum autoantibody levels in lupus-prone mice

To dynamically monitor the incidence of lupus in MRL/LPR mice, our team detected the content of anti-DS-DNA antisubstances and ANA in serum of MRL/LPR mice at each temporal point and in each group via ELISA. In contrast to the controls, the expression levels of sera anti-DS-DNA antisubstance and ANA in model group were remarkably elevated (P < 0.05), which was statistically significant. After GpS treatment, the expression levels of anti-DS-DNA antisubstance and ANA in serum of mice decreased significantly (P < 0.05), this phenomenon suggests that GpS, as a natural plant component, can reduce the production of autoantibodies and slow the progression of SLE, and it is likely to become a new drug for the prevention and remission of SLE (Figure 7).

**Figure 7.** GpS can reduce the level of autoantibodies in the serum of lupus-prone mice. A: ELISA detects the expression level of anti-ds-DNA antisubstance in the serum of MRL/LPR mice in each group at 7, 28, and 56 days (n = 4). B: The ANA expression level in the sera of MRL/LPR mice in every group of 7 days, 28 days, and 56 days was detected by ELISA (n = 4). *P< 0.05.

### GpS can improve kidney function, reduce kidney inflammation and immune complex deposition in lupus-prone mice

We collected urine of MRL/LPR mice at each time point and each group and dynamically detected urinary protein levels to monitor changes in kidney function of MRL/LPR mice after different treatments. The results showed that urinary protein levels increased at different time points and in different groups, and increased gradually with the passage of time (*P*< 0.05). In contrast to the controls, the urine protein level in the model group had a significant increasing trend (*P*< 0.05). In contrast to model group, urine protein level in GpS group showed a decreasing trend in different degrees (*P*< 0.05). In order to study the degree of kidney injury and the deposition of glomerular immune complex and complement in MRL/LPR mice, we carried out immunofluorescence staining to mark IgG and C3 in the kidney, and the outcomes revealed that the deposition levels of IgG and C3 in the model group were greater in contrast to the controls (*P*< 0.05). The outcomes also showed that the fluorescence intensity of IgG and C3 in the kidney tissues of mice in GpS group was remarkably reduced in contrast to model group (*P*< 0.05). (Figure 8)

**Figure 8.** GpS can improve kidney functions in lupus-prone mice, reduce kidney inflammation and immune complex deposition. A: Mouse urine protein level. B: Immunofluorescence detection of IgG deposition in the renal tissues of MRL/LPR lupus mice in each group. C: Immunofluorescence detection of C3 deposition in the renal tissues of MRL/LPR lupus mice in each group. *P< 0.05.

## Discussion

SLE is a common autoimmunity illness, and ULTRAVIOLET light, especially UVB, is the most important environmental factor inducing and aggravating SLE [23]. Autophagy is a common physiological phenomenon in cells, and abnormal autophagy is associated with the onset and progression of many illnesses. Autophagy can be induced by starvation, nutritional deficiency, oxidative stress, ultraviolet radiation, etc. Studies have confirmed that UVB can induce autophagy in cells to varying degrees [24,25].

Gynostemma pentaphyllum is a perennial herbaceous vine of Gynostemma pentaphyllum of Cucurbitaceae, also known as‘“Aescularia chinensi’”,‘“Radix pentaphyllum chinensi’”,‘“Camellia camelli’”, etc. Its main components are GpS, polysaccharide and flavonoids, among which the activity of Gynostemma pentaphyllum saponins has been studied the most [26]. A number of studies have shown that GpS not only has immunomodulatory and anti-inflammatory effects, but also has a unique autophagy regulation effect [27]. Although GpS has extensive efficacy, the molecular mechanism of GpS treatment for SLE is still incomplete. Therefore, the purpose of our study is to explore the specific molecular mechanism of GpS treatment of SLE, so as to explore more targets of GpS in clinical treatment, expand the therapeutic field of GpS, and facilitate the subsequent development of other clinical drugs.

We selected JURKAT cells, an acute T-cell leukemia lineage cell, and induced them with UVB to activate abnormal autophagy. The possible mechanism is that UVB irradiation causes acute light damage to cells, resulting in massive increase of damaged proteins and organelles, and feedback up-regulation of autophagy to maintain the stability of intracellular environment [28]. Inhibition of key proteins bedin-1 and ATG-5 in autophagy will lead to increased apoptosis [29]. Therefore, autophagy can be considered to have a certain protective effect on cell damage caused by UVB and improve cell survival rate, but it also means that damaged cells cannot be cleared in time through the apoptotic pathway, resulting in the accumulation of DNA damage and increasing the risk of cell canceration [30,31]. We found activation of Sirt1/AMPK/mTOR pathway in UVB-induced JURKAT cells. Autophagy can be promoted by AMPK, a critical energy sensor regulating cellular metabolic ability to sustain energy equilibrium, whereas autophagy is inhibited by mammalian mTOR targeting [32]. Sirt1 is also a key protein in the regulation of autophagy. Through sirT1-autophagy pathway, it can relieve the optometritic stress of high fat endoplasm to prevent cirrhosis [33]. Song et al. reported that metformin alleviates hepatosteatosis by restoring SIRT1-mediated autophagy induction via an AMP-activated protein kinase-independent pathway [34]. Moreover, Sirt1 regulates testosterone biosynthesis in Leydig cells via modulating autophagy [35].

In addition, it can inhibit intervertebral disc degeneration by protecting chondrocytes of vertebral endplate from apoptosis and calcification [36,37]. After the addition of GpS, WB outcomes revealed that the phosphorylation of AMPK decreased, the phosphorylation of mTOR increased, the expression of Sirt1 protein decreased, and the activation of the pathway was inhibited. Moreover, autophagy of JURKAT cells was also inhibited. In order to further verify the role of Sirt1 pathway, we activated Sirt1 expression in cells by constructing lentiviral vectors, and the therapeutic effect of GpS was significantly reduced. The above results indicate that GpS can exert autophagy regulation by inhibiting the activity of Sirt1 pathway. To treat SLE.

We further conducted animal experiments to verify the therapeutic effect of GpS on SLE. A large number of apoptotic immune cells in SLE patients gather in the body, which will release a large number of autoantigens, and then induce the activated B cells to produce autoantibodies, presenting lupus-like symptoms [38]. Anti-ds-dna antibody and ANA are important indicators of SLE, and the severity of the disease is significantly positively correlated with these two indicators [39]. Autophagy plays an important role in suppressing auto-inflammation, clearing apoptotic or necrotic cells and immune complexes, and inhibiting the occurrence of lupus-like symptoms [40,41]. The outcomes herein revealed that GpS significantly decreased the level of autoantibodies, alleviated renal inflammation and immune complex deposition, improved renal function, and reduced urinary protein excretion in lupus-prone mice.

The limitation of this study is that the research object is single, and only cell experiments were carried out in vitro. In the future, we need to conduct multi-faceted and all-round studies in humans to demonstrate the effect of GpS on autophagy in multiple pathways related to SLE from both in vivo and in vitro, so as to comprehensively describe the mechanism by which GpS plays a therapeutic role by affecting protein degradation and provide evidence for the treatment of SLE.

## Conclusion

In conclusion, GpS can regulate autophagy and mitochondrial autophagy through Sirt1 pathway, which may be a potential mechanism for GpS to reduce the level of autoantibodies, reduce kidney inflammation and immune complex deposition, improve kidney function, and reduce urinary protein excretion in lupus-prone mice.

## Abbreviations

GpS, gynostemma pentaphyllum saponins; SLE, systemic lupus erythematosus; Sirt1, sirtuin 1; SD, standard deviation; WB, western blotting; CAS, the Chinese Academy of Sciences; FBS, fetal bovine serum; CMU, China Medical University; RT, room temperature; IF, inflammatory factor; MMP, mitochondrial membrane potential.
